# Intelligent Algorithm-Based CT Imaging for Evaluation of Efficacy of Docetaxel Combined with Fluorouracil on Patients with Gastric Cancer

This article has been retracted.

**DOI:** 10.1155/2021/1040374

**Published:** 2021-10-06

**Authors:** Qianqian Chen, Xiaohong Wang, Rong Ding, Ziyao Wang

**Affiliations:** ^1^Department of Gastroenterology, The Affiliated Huai'an Hospital of Xuzhou Medical University and The Second People's Hospital of Huai'an, Huai'an 223002, Jiangsu, China; ^2^Department of CT, The First Affiliated Hospital of Xiamen University, Xiamen 361003, Fujian, China; ^3^Blood Rheumatology and Immunology, Lianshui County People's Hospital, Lianshui County 223400, Jiangsu, China; ^4^Department of Pharmacy, People's Hospital of Hongze District, Huai'an 223100, Jiangsu, China

## Abstract

The study focused on the dual-source computed tomography (CT) images segmented by the decision tree algorithm, to explore the efficacy of docetaxel combined with fluorouracil therapy on gastric patients undergoing chemotherapy. In this study, 98 patients with gastric cancer who were treated in the hospital were selected as the research subjects. The decision tree algorithm was applied to segment dual-source CT images of gastric cancer patients. The decision tree is established according to the feature ring and the segmentation position. The machine inductively learns from the decision tree to extract the features of the CT image to obtain the optimal segmentation boundary. The observation group was treated with docetaxel combined with fluorouracil, and the control group was treated with docetaxel combined with tegafur gimeracil oteracil potassium capsules. The general data of the two groups of patients were comparable and not statistically significant (*P* > 0.05). The two groups were compared for clinical efficacy, physical status, KPS score, improvement rate, and adverse drug reactions after treatment. The results showed that the improvement rate of physical fitness in the observation group was 38.78%, and the improvement rate in the control group was 18.37%. The total effective rate in the observation group was 42.85%, and the total effective rate in the control group was 36.73%. Obviously, the curative effect and improvement rate of physical fitness in the observation group were significantly better than those in the control group (*P* < 0.05). In conclusion, the decision tree algorithm proposed in this study demonstrates superb capabilities in feature extraction of CT images. The machine inductively learns from the decision tree to extract the features of the CT image to obtain the optimal segmentation boundary. The effect of docetaxel combined with fluorouracil is better than that of docetaxel combined with tegafur gimeracil oteracil potassium capsules.

## 1. Introduction

Gastric cancer is a malignant tumor derived from the gastric mucosal epithelium. It ranks second only to lung cancer in mortality among all malignant tumors [1]. Statistics have shown that the prevalence of gastric cancer is increasing year by year. In the early stage, clinical symptoms and signs are antitypical, and approximately 50% of patients have reached the advanced stage when diagnosed. The prognosis of surgery alone is poor, and the 5-year survival rate is only 5%–15%. Therefore, timely and effective treatment of gastric cancer is particularly important [2]. In the last century, great progress had been made in clinical research of gastric cancer in China, but the morbidity and mortality rates are still high. The occurrence of gastric cancer is related to many factors, including living habits, external environmental factors, and diet. It is also related to the differentiation of tissue cells, genetic changes, cell cycle changes, gene expression, and changes in signal transmission pathways [3]. The etiology and pathogenesis of gastric cancer still remain unclear. The early diagnosis rate is low because of a lack of tumor markers that can be used for early diagnosis [4]. Traditional treatment mainly uses fluorouracil or cisplatin, whereas they have large side effects and a low effective rate. The paclitaxel antitumor drugs can act on cell microtubules, block the normal reorganization of microtubules, and stop cells from mitotic division. Docetaxel is a paclitaxel antitumor drug. Studies have shown that docetaxel combined with fluorouracil demonstrates significant effects on gastric cancer patients undergoing chemotherapy [5].

In recent years, CT imaging has been widely used in the clinical diagnosis of gastric cancer, and it shows good results. Dual-source CT is a new device based on mature 64-slice CT technology. It has made a great breakthrough in time resolution, which reaches 83 ms, 0.1 s less than the time required for cardiac imaging. The CT scanning speed is faster than that of heartbeat, which effectively improves the time resolution [6]. There are many ways to segment medical images. The traditional segmentation methods include the area tracking method, the edge detection method, and the threshold method [7]. In recent years, computer-aided diagnosis has achieved good results. Feature extraction based on different algorithms is not only fast but also highly accurate. In the medical field, deep networks are commonly used to extract features to perform pixel classification, and then the candidate frame of the object is processed, but manually distinguishing lesion features is time-consuming and labor-intensive [8].

With the continuous development of intelligent segmentation algorithms, they are often used to learn original images and are extensively used in image segmentation, image classification, and target image positioning [9]. Some scholars have proposed in research that combining pixel information of different scales can extract the best size information [10]. In the study, a decision tree was built based on the feature ring and the segmentation position and then used to extract the features of the CT image to obtain the optimal segmentation boundary, providing a new method for clinical prediction and diagnosis of the occurrence and development of gastric cancer.

## 2. Materials and Methods

### 2.1. Research Subjects

In this study, 98 patients with gastric cancer who were treated in the hospital from February 2018 to February 2021 were selected as the research subjects. The study has been approved by the medical ethics committee of the hospital, and the patients and their families understood the situation of the study and signed an informed consent form.

Inclusion criteria are as follows: (1) patients diagnosed with gastric cancer, (2) patients with no history of chemotherapy, (3) patients with Karnofsky functional status (KPS) score ≥60 points, and (4) patients without language barriers.

Exclusion criteria are as follows: (1) patients with contraindications to CT scan, (2) patients with other mental diseases such as vascular dementia and Lewy body dementia, (3) patients with incomplete clinical data and imaging data, (4) patients with severe liver and kidney dysfunction, (5) patients who were allergic to contrast agents, and (6) breastfeeding or pregnant women.

According to different concentrations of contrast agents, they were divided into the control group and the observation group. In the control group, there were 25 male patients and 24 female patients, with an average age of 58.0 ± 3.2 years. They all had the primary site tumor, including 17 cases of gastric antrum, 10 cases of pylorus, 14 cases of gastric body, and 8 cases of cardia. In the observation group, there were 29 male patients and 20 female patients, with an average age of 57.8 ± 3.4 years. They all had the primary site tumor, including 13 cases of gastric antrum, 15 cases of pylorus, 11 cases of gastric body, and 10 cases of cardia.

### 2.2. Intervention Methods

Before treatment, intelligent algorithm-based CT imaging was performed on the two groups of patients. The observation group was treated with docetaxel combined with fluorouracil. The patient took 7.5 mg dexamethasone tablet orally from the day before administration for consecutive 3 days. On the day of administration, 75 mg/m^2^ docetaxel injection was dissolved in 150 mL of 5% glucose or 0.9% NaCl solution and injected intravenously for 1 hour. 2,400 mg/m^2^ was infected for 5 days from the day of administration. A chemotherapy cycle lasted for 21 days, and at least 2 chemotherapy cycles were required. The control group was treated with docetaxel combined with tegafur gimeracil oteracil potassium capsules. The dosage of docetaxel was the same as that in the observation group. Patients took 80 mg/m^2^ tegafur gimeracil oteracil potassium capsules twice after a meal for 14 days from the day of administration. The treatment cycle was the same as the observation group.

Docetaxel (Jiangsu Hengrui Pharmaceutical Co. Ltd., 0.5 mL specification, batch number: 20100930), fluorouracil (Shanghai Xudong Haipu Pharmaceutical, 10 mg/0.25 g specification, batch number 20101120), and tegafur gimeracil oteracil potassium capsules (Qilu Pharmaceutical Limited company, batch number 140705) were used.

The two groups were compared for short-term clinical efficacy after treatment, physical status after treatment, and adverse drug reactions.

If all lesions disappeared and did not reoccur for 1 month, it was considered a complete remission (CR); if target focal length ≥30% maintained for 1 month, it was considered partial remission (PR); if the total longest diameter of the target lesion increased by 20%, it was considered stable disease (SD), and the sum of CR rate and PR rate was the total effective rate. The toxicity was divided into 0–IV grades as per the grading standard of *Oncology*.

### 2.3. CT Scan

In this study, the Siemens SOMATOM Definition DSCT (Germany) was used to examine the patients. Before scanning, the patients were explained the procedure in detail. The patient was in a supine position, with peripheral venous access to the lower extremity (any lower extremity), and connected to the ECG and blood oxygen monitor. The patient was sedated by a professional anesthesiologist in advance. The dosage of anesthetic used was 2 mL/kg intravenously for 10–15 minutes. At the same time, the patient was observed for electrocardiogram, respiration, and peripheral blood oxygen saturation. The collected CT images were delivered to the workstation, and Functool II software was used to process the images. *Vitrea* version 3.9 was used as the postprocessing workstation.

Dual-source CT scanning was performed. First, the ECG gating technology was used with 80 KV of tube voltage. The tube current parameters were adjusted according to the weight, and the machine automatically gave pitch. The periodic exposure was fully automatic. Unimicron (370 mg I/mL) was used as the contrast agent. MEDRED double-barreled high-pressure syringe was used for the lower extremity vein injection at a flow rate of 0.12 mL/s/kg, and the injection time was 20 seconds. The normal saline was injected at the same flow rate, and the time was 10 seconds.

### 2.4. Inductive Learning Method to Generate Segmentation Boundary

The intelligent algorithm is characterized by machine learning, and a good intelligent system must have good learning capabilities. A constructed segmentation model needs to be optimized by learning to generate the segmentation boundary and formulate the segmentation plan. The inductive learning method can generate the segmentation boundary by selecting the segmentation position. It relies on the inductive reasoning of empirical data. The decision tree is an inductive method based on the Chinese divide-and-conquer algorithm. The tree diagram is used to identify the expected value of each decision plan, and the best decision plan is determined through calculation and reasoning. The structure of the decision tree is generally from top to bottom, and finally different results are obtained, as shown in Figure 1.

Based on the segmentation position of the lesion and the different segmentation point sets, the feature ring decision tree is constructed. The provided feature ring is used to classify and calculate the expected value. The machine intelligent induction learning selects optimized similar features to segment. In this study, the ID3 algorithm is used to inductively learn the decision tree.

If an example set GM has *g* positive examples and *m* negative examples, the ratio of the negative example set ME is expressed as *g*/(*g*+*n*), and the ratio of the positive example set GE is expressed as *g*/(*g*+*n*). The decision tree can be regarded as a message source of the positive and negative sets. Then, the expected value of the message is as follows:

(1) $$\begin{array}{c} I\left(g,n\right)=\frac{g}{g+n}\log_{2}\frac{g}{g+n}-\frac{g}{g+n}\log_{2}\frac{n}{g+n}. \end{array}$$

If the attribute value is *K* = (*k*_1_, *k*_2_, *k*_3_,…, *k*_*r*_), the example set contains *r* subsets (*gn*_1_, *gn*_2_, *gn*_3_,…, *gn*_*r*_).

Let *gn*_*i*_ have *g*_*i*_ positive examples and *n*_*i*_ negative examples, and then the expected value of the subset *gn*_*i*_ is I (*g*_*i*_*n*_*i*_). The weighted mean of the expected values of each subset is the expected value required by the tree rooted at *K*, expressed as follows:

(2) $$\begin{array}{c} E\left(K\right)=\sum_{i=1}^{r}\frac{g_{i}+n_{i}}{g+n}I\left(g_{i}+n_{i}\right). \end{array}$$

The gain of classification information with *K* as the root is as follows:

(3) $$\begin{array}{c} \mathrm{Gain}\left(K\right)=I\left(g,\;n\right)-E\left(K\right). \end{array}$$

Better classification effects of the decision tree indicate larger information gain. The computational complexity of each decision tree node is O((*a*+*m*) × *n*); node is the number of nonleaf nodes; and the computational complexity of the entire algorithm is O((*a*+*m*) × *n* × node). ID3 algorithm is used to process example images. First, the feature ring is extracted for classification. According to the convexity, concavity, completeness, and relative position of the feature ring, a good segmentation boundary generation rule is produced, and then feature rings with identical or similar features are merged to reduce the leaf nodes of the same classification.

### 2.5. Segmentation Boundary Generation

CT images have low contrast, blurred boundaries, and small targets. The size and shape of targets are changeable, and the pixels are close to the blood vessels in the tissue. As a result, it is difficult to distinguish the highly similar features in the CT image, which also increases the difficulty of image segmentation. The feature is optimized based on the inductive learning method, and the boundary is segmented to generate the optimal feature, as shown in Figure 2.

First, the segmentation position is selected, and then the feature ring of the associated features is identified to build a decision tree for induction learning. Feature extraction channels suppress useless features, and useful features generate boundary rules, and finally, segmentation boundaries are generated.

### 2.6. Construction of a Decision Tree

The feature boundary extraction can obtain the end face feature ring and the internal feature ring. Let the feature example set be *H*, *h*_*i*_ is each feature ring, and *T* is the segmentation point set at the selected segmentation position. The Dijkstra shortest path *d*(*hi*) from *h*_*i*_ to the segmentation point *T* is calculated as follows:

(4) $$\begin{array}{c} d\left(hi\right)=\text{Min}\left(d\text{Dijkstra}\left(\varphi_{j},\varphi_{k}\right)\right),\left(\varphi_{j}\in T_{\varphi },\varphi_{k}\in h_{i}\right). \end{array}$$

Dijkstra is a greedy algorithm that selects the optimal solution at each step and obtains the global optimal solution through local optimization.  Figure 3 shows the process to obtain the segmentation boundary. First, the points closest to the segmentation plane are taken to form an edge. If the angle *Q* between the edge and the characteristic surface is within the tolerance value, go to the next step; if not, go back to the first step, and finally, the boundary of the segmentation is obtained using the closure algorithm of the feature ring.

Feature extraction plays an important role in image information classification. CT image information includes mean, median, minimum, maximum, variance, skewness, and kurtosis; image shape features include area, circumference, circularity, elongation, center coordinates of the vertical axis, and center coordinates of the horizontal axis, and shape coefficient; and texture features mainly include contrast, correlation, and entropy.

Mean (*i*-mean) is calculated as follows:

(5) $$\begin{array}{c} \bar{x}=\frac{1}{n}\sum_{i=1}^{n}x_{i}. \end{array}$$

Variance (*i*-std) is calculated as follows:

(6) $$\begin{array}{c} S^{2}=\sqrt{\frac{1}{n}\sum_{i=1}^{n}{\left(x_{i}-\bar{x}\right)}^{2}}. \end{array}$$

Skewness (*i*-skewness) is calculated as follows:

(7) $$\begin{array}{c} D=\frac{1/n\sum_{i=1}^{n}{\left(x_{i}-\bar{x}\right)}^{2}}{{\left(\sqrt{1/n\sum_{i=1}^{n}{\left(x_{i}-\bar{x}\right)}^{2}}\right)}^{3}}. \end{array}$$

*I*-kurtosis is calculated as follows:

(8) $$\begin{array}{c} K=\frac{1/n\sum_{i=1}^{n}{\left(x_{i}-\bar{x}\right)}^{4}}{{\left(1/n\sum_{i=1}^{n}{\left(x_{i}-\bar{x}\right)}^{2}\right)}^{2}}-3. \end{array}$$

Contrast (*t*-contrast) is calculated as follows:

(9) $$\begin{array}{c} A=\sum_{i}\sum_{j}{\left(i-j\right)}^{2}p\left(i-j\right). \end{array}$$

Correlation (*t*-correlation) is calculated as follows:

(10) $$\begin{array}{c} C=\frac{\sum_{i}\sum_{j}{\left(i,j\right)}^{2}p\left(i,j\right)-\mu_{x}\mu_{y}}{\partial_{x}\partial_{y}}. \end{array}$$

Entropy (*t*-entropy) is calculated as follows:

(11) $$\begin{array}{c} E=-\sum_{\text{i}=1}^{L}\sum_{j=1}^{L}p\left(i,\text{j}\right)\log\left(p\left(i,j\right)\right). \end{array}$$

*S*-elongation is calculated as follows:

(12) $$\begin{array}{c} e=\frac{m}{M}. \end{array}$$

Form factor (*s*-form) is calculated as follows:

(13) $$\begin{array}{c} h=\frac{p\times e}{8a}. \end{array}$$

### 2.7. Statistics

The data were processed by SPSS 19.0; the measurement data conforming to the normal distribution were expressed by the mean ± standard deviation ($\bar{x}$ ± *s*); and the nonconforming count data were expressed by the frequency and relative frequency (%). The *t*-test was adopted, the chi-square test was performed for quality comparison, and *P* < 0.05 was the threshold for significance.

## 3. Results

### 3.1. CT Segmentation Results

Figure 4(a) displays CT images of gastric cancer patients. Figures 4(b) and 4(c) explain the imaging images of the selected local features. Figures 4(d), 4(e), and 4(f) show the feature segmentation results. It was noted that the decision tree network can effectively segment the target area in the CT image. The yellow arrow in the figure shows the location of the lesion, and the yellow dashed box represents the range of image feature extraction. Figure 4(a) is the image of a 47-year-old male patient, and it shows the primary site of the tumor was the gastric antrum.  Figure 4(b) is the image of a 58-year-old male patient, and it shows the primary site of the tumor was the pylorus.  Figure 4(c) is the image of a 52-year-old female patient, and it shows the primary site of the tumor was the gastric antrum.

### 3.2. Comparison of Efficacy between the Two Groups of Patients

As shown in Figures 5–7 , there were 3 cases of CR, 18 cases of PR, 19 cases of SD, and 9 cases of PD in the observation group. In the control group, there were 2 cases of CR, 16 cases of PR, 24 cases of SD, and 7 cases of PD. The total effective rate of the observation group was 42.85%, and the total effective rate of the control group was 36.73%. Obviously, the observation group was significantly better than that of the control group.

### 3.3. Comparison of Adverse Drug Reactions

Table 1 shows the adverse reactions of the two groups of patients after taking the drugs. It was noted that the observation group exhibited a lower incidence of leukopenia, nausea and vomiting, thrombocytopenia, hemoglobin reduction, liver impairment, renal impairment, and fever than the control group, and the difference was statistically significant (*P* < 0.05).

### 3.4. KPS Score

Figure 8 shows the KPS score in the two groups. It was noted from Figure 8(a) that the KPS score of the observation group improved in 19 cases, decreased in 6 cases, and stabilized in 24 cases and that in the control group, the KPS score improved in 9 cases, decreased in 22 cases, and stabilized in 18 cases. Figure 8(b) shows that the improvement rate in the observation group (38.78%) was higher than the control group (18.37%), and the difference was statistically significant (*P* < 0.05).

## 4. Discussion

Gastric cancer has high morbidity and mortality rates. Currently, chemotherapy is the main treatment method to maximize the survival period and improve the quality of life of patients. Some anticancer drugs, such as paclitaxel, gemcitabine, and irinotecan, if combined with uracil, have an effective rate of 33%–75% [11]. Docetaxel is a kind of paclitaxel drug, which inhibits the mitosis and proliferation of tumor cells by promoting the assembly of tubulin into stable microtubules [12]. Compared with paclitaxel, docetaxel has a stronger affinity for tubulin and higher antitumor activity, and the residence time in the cell is twice that of paclitaxel [13]. Heath et al. [14] showed that when 75 mg/m^2^ of docetaxel was injected into patients on the first day, the effective rate was 18% and that fluorouracil can effectively interfere with DNA synthesis, and the two demonstrate complementary and synergistic effects. The results of this study showed that the total effective rate of docetaxel combined with fluorouracil was 42.85%, which was significantly higher than the control group. Recently, fluorouracil and its derivatives have been widely used in the treatment of gastric cancer. Fluorouracil has a half-life of 10^−2^ min^−1^. It is a commonly used mid-cell specific drug. Continuous injection of fluorouracil can prolong the inhibition time of thymidylate synthase. Niu et al. [15] found that adjuvant chemotherapy reduces tumor staging, reduces postoperative metastasis and recurrence rates, reduces tumor volume, and effectively increases the removal rate. The results of this study showed that the efficacy of the observation group was significantly better than that of the control group. The total effective rate of the observation group was 42.85%, and that of the control group was 36.73%. The treatment effect of the observation group was significantly higher than that of the control group. Docetaxel combined with fluorouracil has a very good effect.

Intelligent algorithms are widely used to segment CT images. After earning a large number of expert-labeled medical images [16, 17], the machine summarizes the characteristics and rules and finally reaches an expert-level in diagnosis [18]. The artificial intelligence-based pulmonary nodule screening system has shown good results in fracture detection, bone fragility evaluation, and children's bone age evaluation [19, 20]. Chen et al. [21] found that convolutional neural network was used in feature extraction. First, coordinates are generated in the lesion area in the image to generate preselected detection frames, and then the suspicious parts are classified by the trainer. It makes up for the deficiencies of the traditional method of manually extracting the features of the object. The CT image segmented by intelligent algorithms helps accurately detect the location of the lesion, minimize the trauma, and improve the accuracy of diagnosis. In the study, the decision tree is built according to the feature ring and the segmentation position. The machine inductively learns from the decision tree to extract the features of the CT image to obtain the optimal segmentation boundary. In this study, the CT image was segmented by the decision tree algorithm. After induction and learning, the feature extraction channel suppressed useless features, generated boundary rules on the useful boundary, and finally formed the segmentation boundary. Hence, the decision tree algorithm showed a good segmentation effect.

## 5. Conclusion

In the study, an intelligent algorithm was applied to segment dual-source CT images of gastric cancer patients. The decision tree is established according to the feature ring and the segmentation position. The machine inductively learns from the decision tree to extract the features of the CT image to obtain the optimal segmentation boundary. The physical fitness improvement rate of the observation group was significantly higher than that of the control group. The intelligent algorithm proposed in this study demonstrates superb capabilities in feature extraction of CT images, and the effect of docetaxel combined with fluorouracil is better than that of docetaxel combined with tegafur gimeracil oteracil potassium capsules. The limitation of this study is that the sample size is small, and the segmentation of image features cannot reach 100%. In the follow-up, expanded sample size is required to strengthen the findings of the study. In conclusion, the algorithm model of this study can provide a theoretical basis for the extraction of lesion features from CT images in medical systems. In actual applications, CT scanning will be affected by the structure of the scanned object, X-rays, scanning environment, and other factors. CT image reconstruction has high academic value. In future work, more intelligent algorithms are required to elevate the accuracy of the reconstructed images.

## Figures and Tables

**Figure 1:** The decision tree.

**Figure 2:** Schematic diagram of segmentation boundary generation.

**Figure 3:** Flowchart of optimal segmentation boundary.

**Figure 4:** CT image and segmentation results of gastric cancer.

**Figure 5:** The distribution of patients with different efficacy.

**Figure 6:** The efficacy of the two groups of patients.

**Figure 7:** The total effective rate results for the two groups of patients.

**Figure 8:** Comparison of KPS scores between the two groups. Note: ^*∗*^means a statistically significant difference, *P* < 0.05.

**Table 1:** Comparison of adverse conditions between the two groups of patients.

	Adverse reactions	Vomiting	Leukopenia	Thrombocytopenia	Renal impairment	Liver impairment	Fever
Observation group (*N* = 49)	Degree I–II (*n*, %)	11 (22.45)	13 (26.53)	6 (12.24)	7 (14.29)	1 (2.04)	2 (4.08)
	Degree III–IV (*n*, %)	0	3 (6.12)	2 (4.08)	0	0	0
	Total incidence (%)	22.45	32.65	24.32	14.29	2.04	4.08
Control group (*n* = 49)	Degree I–II (*n*, %)	16 (32.65)	16 (32.65)	9 (18.37)	13 (26.53)	3 (6.12)	5 (10.20)
	Degree III–IV (*n*, %)	0	5 (10.20)	3 (6.12)	0	0	0
	Total incidence (*n*, %)	32.65	42.85	24.49	26.53	6.12	10.20

## Data Availability

The data used to support the findings of this study are available from the corresponding author upon request.
